# Comparison of the Effects of Different Testicular Sperm Extraction Methods on the Embryonic Development of Azoospermic Men in Intracytoplasmic Sperm Injection (ICSI) Cycles: A Retrospective Cohort Study

**DOI:** 10.1155/2021/5515247

**Published:** 2021-05-17

**Authors:** Yangyang Hu, Shunshun Cao, Shenghao Wu, Junzhao Zhao, Samuel Kofi Arhin, Dan Shan

**Affiliations:** ^1^Reproductive Medical Center, Department of Obstetrics and Gynecology, The Second Affiliated Hospital and Yuying Children's Hospital of Wenzhou Medical University, Wenzhou, Zhejiang, China; ^2^Endocrinology, Genetics and Metabolism, Department of Yuying Children's Hospital of Wenzhou Medical University, Wenzhou, Zhejiang, China; ^3^Department of Physician Assistant Studies, School of Allied Health Sciences, University of Cape Coast, PMB, Cape Coast., Ghana

## Abstract

**Background:**

The effects of different testicular sperm extraction methods on the embryonic development and clinical outcome of azoospermic men in intracytoplasmic sperm injection (ICSI) cycles have not been researched. Our goal was to evaluate the effect of different sperm retrieval methods used for patients with OA or NOA on the embryonic development and clinical outcomes during the ICSI cycles.

**Methods:**

This was a retrospective cohort study. A total of 530 azoospermic patients who underwent 570 ICSI cycles met the study criteria. ICSI was performed using testicular sperm by TESA in 282 cycles (TESA group); ICSI with testicular sperm by mTESE was performed due to NOA in 90 cycles (mTESE group); ICSI with testicular sperm by MESA was performed in 198 cycles (MESA group). The embryonic development and clinical outcomes of the three groups were counted.

**Results:**

The general characteristics of the three groups were comparable. Our findings showed that the three groups were matched in terms of infertility durations and age. The mean age and the mean BMI of the female partners were similar in the three groups. Also, our findings showed there were no significant differences in the three groups regarding day 3 of the menstrual cycle FSH and days of stimulation. The research results showed that the total dose of FSH and E2 on the HCG administration day was also not statistically different in the three groups. The number of oocytes retrieved had no significant differences in the three groups. However, the number of 2PNs per cycle and the number of cleavages per cycle were higher in the MESA group than in the other two groups; the TESA group and mTESE group were similar. The number of good quality D3 embryos and the number of good quality D5 embryos were significantly decreased in the mTESE group as compared to the other two groups. Good quality D3 embryos and the rate of good quality D5 embryos in the mTESE group were lower than those in the other two groups. Moreover, the clinical pregnancy rates of the TESA group (50.71%) and the MESA group (51.52%) were similar, but both were much higher than that of the mTESE group (32.22%).

**Conclusions:**

The mTESE provides a good clinical outcome for NOA patients with severe spermatogenic impairment, including the rate of good quality D3 embryos, the rate of good quality D5 embryos, and the clinical pregnancy rate. However, our data suggested that both the TESA and MESA groups had better embryonic development and clinical outcomes than the mTESE group.

## 1. Introduction

Over the last three decades, the quality of men's sperm has been decreasing year by year. Azoospermia was defined as semen and urine after ejaculation for 3 consecutive times; no sperm was found by sediment microscopy after centrifugation at >3000 g for 15 minutes (WHO 5th edition). Azoospermia can be divided into obstructive azoospermia (OA) and nonobstructive azoospermia (NOA), of which OA accounts for 40% [1]. Epididymal obstruction is the most common cause of OA. Azoospermia accounts for 1% of the normal population and 10-15% of male infertility [2]. Spermatozoa may be ejaculated in patients with partial OA by vas deferens-epididymal anastomosis. The certain subtypes of azoospermia may be treated with testicular sperm aspiration, following the development of intracytoplasmic sperm injection (ICSI).

Surgical sperm extraction mainly includes percutaneous testicular sperm aspiration (TESA), conventional open testicular sperm extraction (TESE), microsurgical testicular sperm extraction (mTESE), percutaneous epididymal sperm aspiration (PESA), and microsurgical epididymal sperm aspiration (MESA). Different procedures of testicular sperm retrieval were used, mainly based on the etiology (obstructive or nonobstructive) of azoospermia and the surgeon's skills [3]. However, large-scale, well-designed studies of the benefits and safety of one technology relative to another are lacking. The meta-analysis reported a positive sperm extraction rate of 50% in Klinefelter syndrome patients who received mTESE [4]. However, the study observed that the mTESE-positive sperm extraction rate was 21.4% lower than that of the Klinefelter syndrome cohort reported in the meta-analysis [5]. At present, many reproductive centers use mTESE as the preferred method of NOA sperm extraction. Multiple needle-pass TESA is a minimally invasive option and the most commonly used method in clinical practice. The sperm retrieval rate of TESA for NOA was 30%, and that of OA was 100% [2].

With the development of ICSI technology, male infertility has been successfully treated. High pregnancy rates have been reported more and more after treatment of male factor infertility by ICSI. ICSI has been widely used in the world; however, its different sperm sources which affect ICSI clinical outcomes, such as fertilization rate, blastocyst development, implantation rate, and clinical pregnancy rate, have been controversial [4]. A number of studies have reported that the embryonic development of ICSI might be affected by sperm quality, especially in the blastocyst stage [5]. Lee et al. observed that testicular sperm supports embryo development to the blastocyst stage with similar potential as ejaculatory sperm [6].

To date, the clinical efficiency of different testicular sperm extractions in embryonic development and clinical pregnancy rates for azoospermic men have not been researched either at home or abroad. It is not clear whether the source or quality of sperm can affect the embryonic development and clinical outcomes of ICSI. Which testicular sperm extraction in ICSI cycles for azoospermia has the best embryonic development and clinical outcomes? The aim of this study was to compare the clinical efficacy of different testicular sperm extractions in ICSI cycles for azoospermic men and how it happened. Then, we can explore whether one or both meet the clinical requirements and which one is better.

## 2. Materials and Methods

### 2.1. Study Participants

All patients who underwent ICSI cycles with surgical sperm extraction between January 2015 and December 2019 in our in vitro fertilization (IVF) center were candidates for inclusion in this study. The current study was a retrospective study and approved by the ethics committee of the Second Affiliated Hospital of Wenzhou Medical University (Ethic Reference No: L-2020-08). A total of 530 couples who underwent 570 ICSI cycles met the study criteria after exclusion of cases with cryptozoospermia, female infertility, and genetic chromosome abnormality and in whom only ejaculated sperm was used [6]. All male patients were 20~45 years old with infertility due to azoospermia, retrograde ejaculation, and ejaculation difficulties. The women were all under 35 years old. ICSI was performed using testicular sperm by TESA in 282 cycles for 270 couples (TESA group); ICSI with testicular sperm by mTESE was performed due to NOA in 90 cycles for 90 couples (mTESE group); ICSI with testicular sperm by MESA was performed in 198 cycles for 170 couples (MESA group). The embryonic development and clinical outcomes of the three groups were counted. OA and NOA were diagnosed based on physical examination, serum hormone profiling, testicular ultrasound, and three consecutive semen analyses; the blood chromosome was performed in all men. All patients (and family members where applicable) provided written informed consent prior to surgery. All individual operations were performed by the same surgical team. The surgical sperm extraction procedure was performed on the day oocytes were retrieved; thus, fresh testicular sperm was used.

### 2.2. Controlled Ovarian Hyperstimulation (COH) and ICSI Procedure

COH was carried out using a single full-dose injection of 3.75 mg (Triptorelin; Ferring, Kiel, Germany) during the follicular phase of the menstrual cycle. Ovarian stimulation would occur after 32 to 38 days, using recombinant FSH (Gonal-F; Merck Serono, Aubonne, Switzerland). Oocytes were retrieved transvaginally under ultrasound guidance 34~36 h after 5,000~10,000 IU human chorionic gonadotropin (HCG; Livzon, Guangdong, China) injection. After oocyte retrieval, cumulus cells were removed enzymatically and then mechanically for approximately 2 h. Only metaphase II oocytes were fertilized after oocyte retrieval 4~6 h by ICSI. Embryos were incubated at 37°C under humidified and mixed gas (6% CO_2_, 4% O_2_, and 90% N_2_) in and incubator (Labotect C200, Germany). The embryo scores were observed by the same laboratory team under an inverted microscope (Nikon TS100, Japan) [7].

### 2.3. Methodology of the Sperm Retrieval Procedure

#### 2.3.1. Methodology of the TESA Procedure

Disinfect the operating area and lay the operating sheet. Local infiltration of the scrotum was done to anesthetize the scrotum. The surgeon stabilizes the testicle, between the thumb and the index and the middle fingers. The TESA surgery is performed by puncturing an 18-gauge needle into a testicle and applying negative pressure with a 5 ml syringe. Multiple channels run through the testicles. This is done until testicular tissue is visible in the needle. And then, the testicular tissue is immediately put in a Petri dish containing 3 ml of Earle's balanced salt solution. The testicular tissue was then taken to the ART laboratory for investigation. Once spermatozoa were found under the microscope, the operation was terminated [2].

#### 2.3.2. Methodology of the mTESE Procedure

For routine disinfection, lay the operating sheet. The scrotum was then anesthetized by local infiltration. The surgeon stabilizes the testicle. Through a midline incision, the scrotal skin, dartos muscle, tunica vaginalis, and tunica albuginea were opened to expose the testicular tissue. The seminiferous tubules were identified under surgical microscope (Zeiss S88, Germany). Cut out the large seminiferous tubules based on surgical experience. The incised tubules were immediately placed in a Petri dish containing 3 ml of Earle's balanced salt solution. The incised tubules were taken to the ART laboratory for investigation. Then, the testis and scrotum were sutured [8].

#### 2.3.3. Methodology of the MESA Procedure

After disinfection, the surgeon takes a midline scrotal incision or a bilateral transverse scrotal incision. Scrotal skin, dartos muscle, and tunica vaginalis were incised to expose the testis and epididymis. The surgeon fixed the epididymis with the thumb and index finger of the left hand, observed the epididymis under a 10-15 magnification surgical microscope, examined from the tail of the epididymis to the head of the epididymis, and searched and selected those white dilated epididymis tubes, which can usually be found in the head of the epididymis. After the epididymal duct was selected, the tunicae of the epididymis were opened with a microscalpel under a surgical microscope, and the hemostasis was precise by bipolar electrocoagulation. The distended epididymal duct was dissociated with an incision with a diameter of 0.3~0. 5 mm. The epididymis fluid was drawn from the incision with a micropipette and dropped on a sterile slide, and a drop of nutrient solution was added to check the spermatozoa under the microscope.

## 3. Statistical Analysis

The demographic data, age, BMI, serum hormone, embryo data of the three groups were compared. Analysis was performed with SPSS (version 17.0, SPSS Inc., Chicago, USA). ANOVA was used for the comparison of independent samples between three groups if the variance was homogeneous, and Kruskal-Wallis *H* test is used for heterogeneity of variance. Dichotomous variables were analyzed by a chi-square test as required. The data are presented as the mean ± SD. In all analyses, *P* < 0.05 was considered statistically significant.

## 4. Results

The general characteristics of the three groups were comparable. Our findings showed that the three groups were matched in terms of infertility durations (TESA group: 4.01 ± 2.93 vs. mTESE group: 4.39 ± 2.60 vs. MESA group: 4.04 ± 1.90, *P* > 0.05) and age (TESA group: 34.11 ± 4.09 vs. mTESE group: 33.26 ± 3.40 vs. MESA group: 32.36 ± 3.59, *P* > 0.05). The mean age of the female partner (TESA group: 31.48 ± 3.06 vs. mTESE group: 31.17 ± 2.78 vs. MESA group: 29.96 ± 3.50, *P* > 0.05) and the mean BMI of the female partner (TESA group: 22.01 ± 3.64 vs. mTESE group: 21.90 ± 3.29 vs. MESA group: 21.70 ± 3.38, *P* > 0.05) were similar in the three groups. Also, our findings showed that there were no significant differences in the three groups regarding day 3 of the menstrual cycle FSH (TESA group: 5.88 ± 1.68 vs. mTESE group: 6.45 ± 1.80 vs. MESA group: 6.03 ± 1.69, *P* > 0.05) and days of stimulation (TESA group: 11.50 ± 2.40 vs. mTESE group: 11.41 ± 3.04 vs. MESA group: 11.90 ± 2.54, *P* > 0.05). The research results showed that the total dose of FSH (TESA group: 1958.20 ± 723.63 vs. mTESE group: 1795.28 ± 790.34 vs. MESA group: 1865.16 ± 781.08, *P* > 0.05) and E2 on HCG administration day (TESA group: 1995.83 ± 1217.18 vs. mTESE group: 2059.19 ± 1092.63 vs. MESA group: 2085.36 ± 1118.53, *P* > 0.05) were also not statistically different in the three groups. (Table 1).

Table 2 shows that the number of oocytes retrieved (TESA group: 10.67 ± 5.75 vs. mTESE group: 10.09 ± 5.94 vs. MESA group: 11.72 ± 6.25, *P* > 0.05) was not significantly different in the three groups. However, the number of 2PNs per cycle (TESA group: 9.79 ± 5.07 vs. mTESE group: 9.29 ± 5.51 vs. MESA group: 11.00 ± 5.83, *P* < 0.05) and the number of cleavages per cycle (TESA group: 8.56 ± 4.64 vs. mTESE group: 8.03 ± 5.10 vs. MESA group: 9.57 ± 5.38, *P* < 0.05) were higher in the MESA group than in the other two groups; the TESA group and the mTESE group were similar. The number of good quality D3 embryos (TESA group: 6.40 ± 3.43 vs. mTESE group: 3.00 ± 2.76 vs. MESA group: 5.97 ± 3.40, *P* < 0.05) and the number of good quality D5 embryos (TESA group: 2.50 ± 2.25 vs. mTESE group: 1.10 ± 1.27 vs. MESA group: 2.61 ± 2.44, *P* < 0.05) were significantly decreased in the mTESE group as compared to the other two groups. The rate of fertilized eggs (TESA group: 92.51 ± 12.40 vs. mTESE group: 93.32 ± 11.01 vs. MESA group: 94.86 ± 12.82, *P* > 0.05) and rate of cleavage (TESA group: 87.12 ± 14.30 vs. mTESE group: 85.21 ± 18.45 vs. MESA group: 86.06 ± 8.90, *P* > 0.05) were similar in the three groups. The rate of good quality D3 embryos (TESA group: 77.69 ± 17.55 vs. mTESE group: 38.98 ± 28.96 vs. MESA group: 66.02 ± 19.21, *P* < 0.05) and the rate of good quality D5 embryos (TESA group: 27.36 ± 20.72 vs. mTESE group: 12.08 ± 14.21 vs. MESA group: 25.30 ± 20.55, *P* < 0.05) in the mTESE group were lower than those in the other two groups. Moreover, the clinical pregnancy rates of the TESA group (50.71%) and the MESA group (51.52%) were similar, but both were much higher than the mTESE group (32.22%). The rate of sperm retrieved for the TESA group (92.16%) and the MESA group (88.79%) was higher than that of the mTESE group (51.14%) (Table 2).

## 5. Discussion

In the past few years, growing interest has been paid to predicting the sperm retrieval rate and pregnancy rates in azoospermic men, who underwent mTESE, but the results remain inconsistent. Çayan et al. reported a study that NOA men with a history of cryptorchidism have high sperm retrieval rates with mTESE [9]. However, some studies have shown that there are no precise and noninvasive methods for predicting whether there are testicular spermatozoa in NOA patients before mTESE [10]. Maglia et al. found that the success rate of sperm retrieval in NOA patients was similar between the mTESE group and the conventional TESA group, and mTESE seemed to be more beneficial for patients over 35 years of age and with high FSH value [11].

Up to now, what these previous studies had in common was a prediction of sperm retrieval rate [12]. The clinical efficiency of different testicular sperm extractions on the embryo development and clinical pregnancy rates of azoospermic men have been rarely reported. In our study, the rate of good quality D3 embryos and the rate of good quality D5 embryos in the mTESE group were lower than those in the other two groups. Our data simultaneously showed that the clinical pregnancy rate in both the TESA group and the MESA group were higher than that in the mTESE group. It may be related to the difference in the quality of sperm obtained by different sperm retrieval groups. mTESE is mainly used in patients with NOA while TESA and MESA are mainly used in patients with OA. MESA is most commonly used in azoospermic patients with epididymal obstruction. In NOA patients, testicular spermatogenesis was only focal, while in OA patients, testicular spermatogenesis was almost normal.

A prospective study by Cito et al. revealed that the reactive oxygen species (ROS) production of NOA was significantly higher than that of normozoospermic men, and it may be related to spermatogenesis disorders in NOA patients [13]. Vatannejad et al. published a study revealing that ROS also damage sperm nuclear DNA, displaying a negative effect on sperm DNA fragmentation [14]. Some studies have shown that compared with the epididymis or testicular sperm of OA patients, the fertilization rate, clinical pregnancy rate, and delivery rate of NOA patients were lower in ICSI cycles [15–17]. Tesarik published a study revealing that NOA patients with severe spermatogenesis impairment are more likely to have testicular sperm defects, such as those associated with centrioles and genetic material, that ultimately affect the ability of the male gamete to activate the egg and development of zygotes and embryos [18]. It also confirms our results that the sperm quality of NOA is significantly lower than that of OA.

Our data simultaneously showed that the rate of good quality D3 embryos, the rate of good quality D5 embryos, and the clinical pregnancy rate both in the TESA group and in the MESA group were similar. A prospective study by Weng et al. demonstrated that chromosomal aneuploidy was similar in azoospermic men who required MESA or TESA for ICSI [19]. In 2011, Keltz et al. found that in patients undergoing TESA-ICSI cycle failure, a repeat cycle with MESA-ICSI may result in marked improvement in outcome [20].

## 6. Conclusions

In conclusion, mTESE provides a good clinical outcome for NOA patients with severe spermatogenic impairment, including the rate of good quality D3 embryos, the rate of good quality D5 embryos, and the clinical pregnancy rate. However, our data suggested that both the TESA and MESA groups had better clinical outcomes than the mTESE group. With these fundamental data, the study could provide a reference for the selection of the appropriate methodology of the sperm retrieval and ICSI treatment.

## Figures and Tables

**Table 1:** Couples' basic characteristics of the three groups.

	TESA group	mTESE group	MESA group	*P*
No. of couples	270	90	170	
No. of cycles	282	90	198	
Infertility durations (years)	4.01 ± 2.93	4.39 ± 2.60	4.04 ± 1.90	0.06
Age (years)	34.11 ± 4.09	33.26 ± 3.40	32.36 ± 3.59	0.12
Age of female partner (years)	31.48 ± 3.06	31.17 ± 2.78	29.96 ± 3.50	0.26
BMI of female partner (kg/m^2^)	22.01 ± 3.64	21.90 ± 3.29	21.70 ± 3.38	0.86
Day 3 of the menstrual cycle FSH (IU/l)	5.88 ± 1.68	6.45 ± 1.80	6.03 ± 1.69	0.23
Days of stimulation (days)	11.50 ± 2.40	11.41 ± 3.04	11.90 ± 2.54	0.17
Total dose of FSH (IU)	1958.20 ± 723.63	1795.28 ± 790.34	1865.16 ± 781.08	0.15
E2 on hCG administration day (pg/ml)	1995.83 ± 1217.18	2059.19 ± 1092.63	2085.36 ± 1118.53	0.70

**Table 2:** Laboratory and clinical outcomes of the three groups.

	TESA group	mTESE group	MESA group	*P*
No. of oocytes retrieved	10.67 ± 5.75	10.09 ± 5.94	11.72 ± 6.25	0.06
Rate of sperm retrieved (%)	92.16 (282/306)	51.14 (90/176)	88.79 (198/223)	
No. of 2PNs per cycle	9.79 ± 5.07	9.29 ± 5.51	11.00 ± 5.83	0.02
No. of cleavage per cycle	8.56 ± 4.64	8.03 ± 5.10	9.57 ± 5.38	0.04
No. of good quality D3 embryos	6.40 ± 3.43	3.00 ± 2.76	5.97 ± 3.40	<0.01
No. of good quality D5 embryos	2.50 ± 2.25	1.10 ± 1.27	2.61 ± 2.44	<0.01
Rate of fertilized eggs (%)	92.51 ± 12.40	93.32 ± 11.01	94.86 ± 12.82	0.14
Rate of cleavage (%)	87.12 ± 14.30	85.21 ± 18.45	86.06 ± 8.90	0.44
Rate of good quality D3 embryos (%)	77.69 ± 17.55	38.98 ± 28.96	66.02 ± 19.21	<0.01
Rate of good quality D5 embryos (%)	27.36 ± 20.72	12.08 ± 14.21	25.30 ± 20.55	<0.01
Clinical pregnancy rate (%)	50.71 (143/282)	32.22 (29/90)	51.52 (102/198)	

## Data Availability

The data used to support the findings of this study are available from the corresponding author upon request.
